# Leptomeningeal carcinomatosis from renal cell cancer: treatment attempt with radiation and sunitinib (case report)

**DOI:** 10.1186/1477-7819-8-36

**Published:** 2010-05-05

**Authors:** Astrid Dalhaug, Ellinor Haukland, Carsten Nieder

**Affiliations:** 1 Department of Oncology and Palliative Medicine, Nordland Hospital, Bodø, Norway; 2 Faculty of Medicine, Institute of Clinical Medicine, University of Tromsø, Tromsø, Norway

## Abstract

A case of leptomeningeal carcinomatosis in a patient with known brain and lung metastases from renal cell cancer without previous systemic therapy is presented. Neoplastic meningitis (NM) developed 31 months after first diagnosis of simultaneous extra- and intracranial recurrence of kidney cancer and surgical resection of a cerebellar metastasis. In spite of local radiotherapy to the macroscopic NM lesions in the cervical and lumbar spine followed by initiation of sunitinib, the patient succumbed to his disease 4 months after the diagnosis of NM. The untreated lung metastases progressed very slowly during almost 3 years of observation. This case illustrates important issues around both biological behaviour and treatment approaches in metastatic renal cell cancer.

## Background

Brain metastases from renal cell carcinoma might develop many years after primary nephrectomy and continue to represent a formidable challenge [1]. With increasing numbers of local and systemic treatment options, the issue of patient selection gains importance. While surgery and stereotactic radiosurgery (SRS) provide long-term local control of macroscopic disease, development of new central nervous system lesions can often be observed. Some patients might even present with leptomeningeal carcinomatosis or so called neoplastic meningitis (NM). Only few cases of NM from renal cell carcinoma treated with contemporary systemic approaches have been reported [2,3]. Therefore, the present case illustrates important aspects around potential treatment options.

## Case presentation

A 72-year-old male presented to his family doctor with a 3 week history of headache and dizziness. His medical history was unremarkable except for left-sided nephrectomy for clear cell renal cell cancer stage T2 N0 M0 8 years earlier. Diagnostic imaging with brain computed tomography (CT) scan followed by magnetic resonance imaging (MRI) revealed a 3 cm large contrast-enhancing infratentorial tumor (Figure 1). No additional brain lesions were detected. CT of chest and abdomen revealed 2 small lung nodules (one left-sided, one right-sided) and enlarged mediastinal lymph nodes (Figure 2). Neurosurgical resection of the intracranial tumor confirmed metastasis from clear cell carcinoma. Neither postoperative radiotherapy nor systemic treatment was recommended at this time. Surveillance CT scans showed very slow enlargement of the lung and lymph node metastases during the next year. Seventeen months after resection of the cerebellar metastasis, local recurrence was detected. The patient was treated with gamma knife SRS (peripheral dose 21 Gy). Six months later, a single new brain metastasis was found (8 mm large, left occipital lobe), which also was treated with SRS. Seven months after the second SRS procedure, a third one was added after diagnosis of two new infratentorial brain lesions (cerebellum and brain stem, respectively). Treatment planning MRI also revealed a contrast-enhancing extramedullary mass at the level of the 5th cervical vertebra. Additional scans of the spine showed at least two more small metastases in the lower thoracic and upper lumbar region (Figure 3). No cerebrospinal fluid (CSF) examination was performed as imaging and history were consistent with a diagnosis of NM. The involved regions were treated with fractionated external beam radiotherapy (10 fractions of 3.5 Gy). At that time, the patient had a Karnofsky performance status (KPS) of 70. He had no new focal neurologic deficits, but continued to experience dizziness and gait disturbance since his first SRS procedure. Because of intense pain in different skeletal regions, a radioisotope bone scan was performed, which showed bone metastases in the corresponding areas. These metastases were confirmed by radiographs and/or CT. Analgetic treatment with opiods was started and external beam radiotherapy fields were added to parts of the pelvis, femur and shoulder. For the first time during follow-up, elevated lactate dehydrogenase levels (266 U/L) and lymphopenia (0.3 × 10^9^/L) were seen. The known lung and lymph node lesions continued to progress slowly (Figure 2). Three weeks after radiotherapy, the first systemic treatment was initiated, consisting of sunitinib 50 mg per day. After two weeks on sunitinib, the patient presented to the emergency room with chills and reduced general condition. Fever (38.7°C), elevated C-reactive protein (CRP) level (235 mg/L), leukopenia (3.2 × 10^9^/L) and thrombopenia (73 × 10^9^/L) were found. Blood- and urine cultures were negative. Chest X-ray showed a small infiltrate. Sunitinib treatment was stopped and antibiotic therapy initiated. The patient recovered, but was still unable to reduce analgesics and had a KPS of 50. The treating oncologists decided to stop active cancer treatment. Three weeks later, he began to lose strength in the lower extremities. Steroid treatment was unsuccessful. Imaging was not repeated as management would not have been altered. Another three weeks later, the patient again presented to the emergency room with chest pain, dyspnea and tachycardia. Chest X-ray revealed pneumonia, CRP was elevated to 228 mg/L, leukocyte counts normal (6.6 × 10^9^/L). In spite of antibiotic treatment, the patient succumbed to his disease a few hours after admission. Survival was 11 years from nephrectomy, 35 months from initial diagnosis of brain and lung metastases, and 4 months from NM and bone metastases.

**Figure 1:** **Preoperative T1-weighted magnetic resonance imaging showing a 3 cm large contrast-enhancing infratentorial tumor**.

**Figure 2:** **Computed tomography of the chest showing mediastinal lymph node enlargement (upper image: September 2005, i.e. initial diagnosis of metastases)**. Slow progression in the absence of treatment (lower image: June 2008, i.e. before initiation of sunitinib therapy). The white arrow indicates metastasis in a thoracic vertebra.

**Figure 3:** **Magnetic resonance imaging (T1-weighted post Gadolinium) showing two of several contrast-enhancing leptomeningeal metastases, indicated by white arrows**.

## Conclusions

NM from renal cell carcinoma is a rare event, with only few cases reported to date [2,3]. In the present patient, it was preceded by brain metastases, initially a single cerebellar lesion, which was surgically removed. Whether resection of posterior fossa metastases increases the risk of leptomeningeal dissemination is a topic of debate. Recent data suggest that en bloc removal of metastatic lesions does not increase the risk [4]. Fractionated external beam radiotherapy might offer symptom palliation in patients with brain metastases from kidney cancer [5]. Median survival was 3 months. Median survival and long-term survival rates are higher in patients treated with surgical resection or SRS. In a series of 32 patients, SRS resulted in median survival of 10 months and 3-year survival of 16% [6]. A large analysis including more than 1000 patients treated with SRS without additional whole-brain radiotherapy (WBRT) showed that approximately 50% developed new lesions (several types of primary tumors were included) [7]. Comparable findings were made in surgery series. The addition of WBRT to either SRS or surgical resection decreased the in-brain failure rates but failed to improve survival, most likely because new lesions can be treated with salvage SRS or surgery [8-10]. It has been argued that delaying WBRT may be appropriate for some subgroups of patients with SRS-treated brain metastases from renal cell carcinoma and other relatively radioresistant tumors [11]. As these subgroups are not well defined, individual discussion and decision is necessary. In the present case, no postoperative radiotherapy was administered. Instead, salvage SRS was given to the sites of intracranial relapse. A previous study included analyses of the impact of systemic treatment on survival. Systemic immunotherapy with interleukin-2 and interferon was associated with improved 3-year survival, while treatment with antiangiogenic agents was not [6]. Nevertheless, antiangiogenic agents have become a mainstay of treatment in the general population of patients with metastatic renal cell carcinoma and occasional responses of brain metastases to these drugs have been reported [12]. In another series with 138 renal cell carcinoma patients with brain metastases, 5-year survival was 12% [13], suggesting that aggressive management should be considered in prognostically favorable patients.

Surgical resection should be considered in patients with renal cell carcinoma developing metachronous lung metastases [14], but in the present case bilateral lesions and mediastinal lymph node metastases were detected. In addition, the diagnosis of brain metastasis argued against lung surgery. The untreated lung and lymph node lesions progressed very slowly (Figure 2), a finding not uncommon in this disease. Nevertheless, these metastases might have been the source of further dissemination. The slow growth rate and absence of clinical symptoms prompted the treating oncologists to postpone systemic therapy. This decision was also influenced by the potential serious toxicity of systemic therapy. If tailored to the clinical symptoms, systemic therapy would not have been necessary before the almost simultaneous detection of leptomeningeal and bone metastases. However, at that time careful consideration of treatment options was necessary. It was felt that radiotherapy to the macroscopic spinal lesions was more appropriate than to the complete craniospinal axis, both with regard to reduced bone marrow toxicity and treatment time. The aim was to avoid delays in systemic therapy or reduced doses because of neutro- and/or thrombopenia. Intrathecal chemotherapy should be considered in patients with NM from breast cancer or hematologic malignancies. In patients with renal cell carcinoma, its role is less well defined.

Sunitinib, which is currently used as first-line treatment in patients with metastatic renal cell carcinoma in Norway, resulted in median progression-free survival of 10.8 months in a large trial where 375 patients received the drug [15]. Its role in patients with limited performance status and/or central nervous system metastases is not well defined and requires additional studies. We are not aware of clinical data supporting its use in patients with NM. The patient presented here developed both hematologic and infectious complications after 2 weeks on sunitinib and treatment was then discontinued. In addition, the patient's general condition deteriorated slowly. Eventually, he died from pneumonia. Survival after NM was 4 months. This figure is comparable to data in mixed patient groups (breast cancer, lymphoma, lung cancer etc.), where those with KPS 70 or greater had median survival of 15.5 weeks and those with KPS <70 only 6 weeks [16]. The presence or absence of CSF cytology did not influence survival [17]. Overall, NM is often associated with extensive extracranial disease burden and short survival in spite of treatment with radio- and chemotherapy [18]. Performance status and extent of disease should guide the choice of treatment [19]. Studying the role of renal cell carcinoma-specific systemic treatment approaches requires collaborative efforts because NM is a rare event is this particular disease.

## Competing interests

The authors declare that they have no competing interests.

## Authors' contributions

CN, EH and AD collected patient data and follow-up information. CN and AP drafted the manuscript. All authors read and approved the final manuscript.

## Consent

Written informed consent was obtained from the patient's relative for publication of this case report and any accompanying images. A copy of the written consent is available for review by the Editor-in-Chief of this journal.
